# Analysis Model of Image Colour Data Elements Based on Deep Neural Network

**DOI:** 10.1155/2022/7631788

**Published:** 2022-07-18

**Authors:** Chao Jiang, Zhen Jiang, Daijiao Shi

**Affiliations:** School of Arts, Anhui University of Finance and Economics, Bengbu 233030, Anhui, China

## Abstract

At present, the classification method used in image colour element analysis in China is still based on subjective visual evaluation. Because the evaluation process will inevitably be disturbed by human factors, it will not only have low efficiency but also produce large errors. To solve the above problems, this paper proposes an image colour data element analysis model based on depth neural network. Firstly, intelligent analysis of image colour data elements based on tensorflow is constructed, and the isomerized tensorflow framework is designed with the idea of Docker cluster to improve the efficiency of image element analysis. Secondly, considering the time error and spatial error diffusion model in the process of image analysis, the quantization modified error diffusion model is replaced by the original model for more accurate colour management. Image colour management is an important link in the process of image reproduction; the rotating principal component analysis method is used to correct and analyze the image colour error. Finally, using the properties of transfer learning and convolution neural network, an image colour element analysis model based on depth neural network is established. Large-scale image data is collected, and the effectiveness and reliability of the algorithm are verified from different angles. The results show that the new image colour analysis method can not only reveal the true colour components of the target image; furthermore, the real colour component of the target image also has high spectral data reconstruction accuracy, and the analysis results have strong adaptability.

## 1. Introduction

Traditional colour matching is limited by specific conditions [1]. Once the environmental factors of cie-d65 light source and 1931 standard observer change, the matching effect will be affected accordingly [2]. This conditional matching method usually leads to the phenomenon of homochromatic spectrum [3]. Therefore, this paper proposes an ideal spectrum matching method (or unconditional colour matching), which is the theoretical basis of the accurate colour reproduction technology based on spectrum [4]. In order to realize the ideal spectral matching method, we must first determine a group of basic colour components to represent and reproduce the original colour in multispectral space [5]. That is, the spectral information of the original image can be accurately reconstructed through the linear combination of several prediction components in the linear colour mixing space. The only clue to produce the above prediction components is a set of eigenvectors obtained from the corresponding spectral measurement data and principal component analysis. Image restoration is one of the most important and basic fields of image processing, which has important theoretical value and practical significance [6]. In the process of image capture, transmission, and conversion, it will inevitably cause image degradation. The typical manifestations are image blur, distortion, and noise. In the further application of images, such as feature extraction, automatic recognition of terrain and fingerprint, and image data analysis, clear and high-quality images are needed. Therefore, in many fields such as aerospace, medicine, military public security, and image coding, in order to suppress noise and improve image quality, it is of great practical significance [7]. An important problem to be solved in image processing is how to restore the original image reflecting the real scene of the objective world with the observed image as the known data. There are many reasons for image degradation, which can be roughly divided into deterministic factors and random factors. The deterministic factors include improper focusing of the imaging system, the relative motion between the imaging equipment and the target object, and the defects of the imaging system itself, as well as the atmospheric turbulence effect that needs to be considered in long-time exposure [8]. On this basis, many scholars have developed many improved methods, such as restraining noise and protecting edges by introducing constraints.

Randomness factor mainly refers to the noise pollution of image signal in the process of transmission, digitization, and recording. Image restoration is to use the prior knowledge leading to image degradation to establish the mathematical model of image degradation, and then restore along the inverse process of image degradation to obtain a clear original image. The difficulty of restoration mainly depends on the mastery of the prior knowledge of the degradation process. The traditional image restoration methods can be roughly divided into inverse filtering method, algebraic method, and spatial filtering method. On this basis, many scholars have successively studied many improved methods, such as restraining noise and protecting edges by introducing constraints [9]. This method is van cittert iteration of image restoration with fuzzy smoothing constraints [10]. For image processing, the amount of calculation of iterative algorithm is very large. Convergence speed is also an important index to measure its performance; in order to overcome the limitation of restoring a clear scene from a single image, literature [11] proposes a method based on polarized light by using multiple images or additional information. This method requires that the scene and camera do not change when multiple images are taken, so it is difficult to be used in dynamic scenes. In literature [12], it is necessary to collect multiple images of the same scene under different weather conditions. This method can effectively restore the image contrast, but it cannot deal with unknown scenes and dynamic scenes. Literature [13] proposed a smoothing constraint based on the edge direction criterion. The regularization operator obtained by this method can suppress the noise and protect the image edge information at the same time [14]. However, in the case of serious image degradation, the flat area of the image is easy to be misjudged as the edge area. One result is that the existence of artefacts in the restored image cannot be estimated accurately [15].

Principal component analysis is a commonly used multivariate statistical method, which is very effective in information compression and data correlation elimination. It has been widely used in face, license plate, and other feature extraction. In recent years, some researchers have applied principal component analysis to colour science [16]. Literature [16] proposed a colour prediction scheme based on PCA, which can estimate a group of basic colour components that can most accurately restore the original image according to a large number of colour samples. However, when the principal component analysis method based on K-L transformation is directly used to obtain the feature vector corresponding to the undetermined colour component, “negative index” problem appears [17]. According to the statistical properties of principal component analysis, except that the positive and negative of the first eigenvector can be correctly judged, the positive and negative of other eigenvectors are often difficult to judge, and the smaller the variance in the direction of the eigenvector, the harder it is to judge the positive and negative. In other words, the first principal component can judge whether it is a positive indicator according to the positive and negative of the coefficient (i.e. eigenvector) corresponding to the original variable, while the coefficient symbols corresponding to each original variable in other principal components are often inconsistent. At this time, the principal component is recognized as a negative indicator. It can be seen that the problem of “negative index” in K-L transformation depends on the positive and negative judgment of eigenvector. The relationship between the undetermined colour component and the corresponding feature vector can be determined by some linear transformation or geometric rotation. The black box rule is to regard the whole as a black box without considering the factors related to the equipment in the colour conversion, only analyze and fit the input and output colour values of a certain number of standard colour blocks, and then interpolate the spatial relationship to obtain the conversion relationship of other colour blocks [17]. Such methods include Neugebauer equation method, one-dimensional nonlinear function method, linear or matrix conversion method, multidimensional table conversion method and polynomial fitting algorithm, and the transformation method based on BP network [18] and machine learning [19]. Because the black box method does not consider the intermediate process of colour conversion and only controls the input and output values, it is difficult to ensure the conversion accuracy. In literature [20, 21], it is necessary to collect multiple images of the same scene under different weather conditions. This method can effectively restore the contrast of the image, but it cannot deal with unknown scenes and dynamic scenes. Reference [22] proposed a smoothing constraint based on the edge direction criterion. The regularization operator obtained by this method can suppress noise and protect the edge information of the image. However, in the case of serious image degradation, the flat area of the image is easy to be misjudged as an edge area, resulting in the inability to accurately estimate the existence of artifacts in the restored image. To solve the above problems, this paper proposes an image colour data element analysis model based on neural network.

## 2. The Intelligent Analysis of Image Colour Data Elements Based on Tensorflow

### 2.1. The Structure Design of Intelligent Analysis of Image Colour Data Elements

The corresponding application modules are developed and implemented on the Android mobile device platform [23]. Its development environment mainly includes the following: Taking Java 8.0, which can operate across platforms, as the development language; Take Android studio 2.1.3 as the development integration environment; Take Android SDK 23 as the target version. The system includes three modules: image element recognition module, image element knowledge module, and image element information storage module. The deep learning model is retrained by using the transfer learning method and the image data with enhanced texture features. Combined with the convolution neural network, the image colour element analysis model is established, and the overall structure is shown in Figure 1. The image element recognition module is divided into two parts: real-time photo recognition and local library recognition, with the coupling model as the core; the knowledge module of image elements includes physical properties and uses; the image element information storage module is divided into two parts: image basic information storage and additional information storage. The knowledge card module is the main module of the system, which provides the functions of real-time identification of mobile camera and local album identification. The recognition result interface is the link of the system and can be linked to the knowledge card module and mobile phone storage module. In the recognition result interface, the interaction function can be realized according to the recognition result and the relevant information in the knowledge card; by editing the text box, the picture and text information can be saved in the data storage module.

The identification module can be divided into two submodules: photo identification and local album identification. The process of local album recognition is basically the same as that of photo recognition. The original image is saved and displayed in the result interface according to the type of recognition. Photo recognition is real-time recognition. Field workers can adjust the focal length and position of the camera according to their own needs and the shape of minerals so as to obtain multiple recognition results for the same image. At the same time, the function of real-time recording is also added in the recognition result interface. Mobile phone local album identification can prevent identification omission. The identification application can sort out photos stored locally by reading them. Knowledge card module: the knowledge card module interface is the home page of the application system. By comparing the application recognition results with the nature of the images recorded in the knowledge card, field workers can more accurately judge the types of image elements. Data storage module: the information storage module is developed based on the identification module. Its storage mode is divided into three levels based on the timeline and identification results. The root directory is named after the photographing date, and the subdirectories under the root directory are named after the recognized types. Finally, the pictures are stored in the recognition result directory and named by hours and minutes and seconds, respectively. At the same time, with the increase of the number of stored pictures, the dataset of model training continues to increase, and it can be continuously used for the retraining of the recognition model and finally improve the model accuracy and recognition accuracy.

### 2.2. Design of Isomerization Tensorflow Architecture Based on Docker Container Cluster

Docker adopts the standard C/S architecture mode, which is divided into two parts: client and server. The Docker client creates and manages the Docker container by establishing communication with the Docker daemon, which receives and processes requests from the Docker client. The structural diagram of isomerized tensorflow is shown in Figure 2. In terms of design, Docker server is a very loosely coupled architecture. Each module has a clear division of labor and combines with each other to jointly support the operation of Docker. Docker customizes the Docker container running environment through the driver module. When you need to create a Docker container, you can download the relevant image from the Docker registry and store the relevant image locally in the form of graph through the graphdriver. When the Docker container needs to create a network, you can use the networkdriver to create and configure the network environment for the Docker container; using execdriver, you can limit Docker container resources or execute relevant instructions. Networkdriver and execdriver realize the actual operation of containers through independent container management file libcontainer, including using namespace subsystems such as file system, network, PID, UID, and IPC to isolate each container and using CGroup to limit the resource allocation of containers. After the command to run the container is executed, a Docker container with independent file system and isolated environment will be running. Tensorflow is not only an interface to implement deep learning algorithm but also a framework to execute deep learning algorithm. It plans the whole computing process through data flow diagram and can map different computing modules to a variety of computing devices and platforms. With its unified architecture, it can be easily transplanted over many heterogeneous systems, which greatly simplifies the application difficulty of deep learning in the real scene.

By deploying tensorflow in the Docker container to isolate and restrict the underlying resources, tensorflow is virtualized and heterogeneous so as to obtain high portability on multiplatform and multisystem. Through the design of elastic container cluster system architecture, realize the distributed deployment of tensorflow deep learning system and improve the data throughput of the platform; on this basis, the parallel training of neural network is realized through two different schemes of data segmentation and model segmentation so as to solve the problem of long time of deep learning training.

## 3. The Design of Analysis Model of Image Colour Data Elements Based on Deep Neural Network

Using the transfer learning method, the depth learning model is retrained by using the image data with enhanced texture features, and the colour model of image recognition is established by using k-means. Finally, the coupling model of image recognition is established. The overall method structure is shown in Figure 3. The image element coupling model is coupled by the retraining concept-v3 model and the colour model. In the recognition process, firstly, the heavily trained perception-v3 model is used to classify the enhanced texture image, and then the image is input into the colour model so that the final recognition result is output from large to small according to the probability obtained by the coupled recognition analysis model.

Under illumination conditions, different images have different reflection degrees of light, and the same cleavage surface has regular change characteristics. Therefore, the brightness and colour also show corresponding regular changes in the image, so the texture features can be extracted according to the brightness and colour changes of the cleavage surface in the image. Extracting the brightness change area in the image and depicting it with lines can achieve the effect of image feature extraction. The image is a colour image. Therefore, based on the colour space theory, the RGB value of each pixel can be extracted from the image, and the gray value of each pixel is calculated by the following formula:

(1) $$\begin{array}{c} \text{Gray}=0.229\times R+0.587\times G+0.114\times B, \end{array}$$

where Gray is the gray value of the pixel; *R*, *G*, and *B*, respectively, correspond to the three primary colour values of pixels. Under the illumination condition, the brightness change of the image texture part will be significantly different from the illumination change of the surrounding pixels. In the texture part, the gray value of the image increases or decreases sharply. Therefore, the image texture information can be extracted by brightness change.

(2) $$\begin{array}{c} \Delta Z_{i}={\text{Gray}}_{i}-\left\{\sum_{i=1}^{n=9}{\text{Gray}}_{i}-{\text{Gray}}_{\max}-{\text{Gray}}_{\min}\right\}, \end{array}$$

where Δ*Z*_*i*_ is the brightness change value of the pixel; Gray is the gray value of the pixel, which is determined by formula (2); In order to eliminate the possible boundary interference, the maximum (Gray_max_) and minimum (Gray_min_) in the gray value are removed.

(3) $$\begin{array}{c} {\left|\Delta Z_{i}\right|}^{\prime }=\left|\Delta Z_{i}\right|-\left|\Delta \bar{Z}\right|, \end{array}$$

where | |Δ*Z*_*i*_|′ is the change of gray value at point *i*; Take *T* as the threshold value, and take the maximum value of the absolute value of the brightness value difference. When the change value of pixel illumination is less than the threshold, it is not set as a feature point; when the brightness change value is greater than the threshold value, it is set as the feature point. The test shows that when *t* = 15, the image feature extraction effect is good.

### 3.1. Image Colour Analysis Algorithm Based on Error Diffusion Model

In the process of image processing, error correction is required. The colour information transmission between different devices, the conversion of different colour gamut spaces, and the colour errors are all managed through error correction. The quantization corrected error diffusion model is replaced by the original model for more accurate colour management.

Error diffusion can be divided into space error diffusion and time error diffusion. At the same time, pixel error diffusion can be divided into left error diffusion and right error diffusion. The separable error diffusion framework is shown in Figure 4. One pixel position *p*(*x*, *y*, *z*), the image brightness is *I*(*x*, *y*, *z*), and the adjacent point of the pixel is *ε*(*x*, *y*, *z*). Quantized into *I*_*d*_(*x*, *y*, *z*), and the quantization error is *T*(*x*, *y*, *z*) through threshold comparison

(4) $$\begin{array}{c} \left\{\begin{array}{c} \hat{I}\left(x,y,z\right)=I\left(x,y,z\right)+\varepsilon \left(x,y,z\right),\\ I_{d}\left(x,y,z\right)=\left\{\begin{array}{cc} 1, & \text{otherwise,}\\ 0, & I\left(x,y,z\right)+\varepsilon \left(x,y,z\right)<T\left(x,y,z\right). \end{array}\right. \end{array}\right. \end{array}$$

The time error diffusion formula is

(5) $$\begin{array}{c} \left\{\begin{array}{c} g_{t}\left(x\right)=\exp\left\{-{\left(\frac{\ln\left(t/\tau \right)}{\sigma }\right)}^{2}\right\},\\ \lambda_{t}\left(x,y,z\right)=1-\exp\left\{-\frac{{\left(I\left(x,y,z\right)-\hat{I}\left(x,y,z\right)\right)}^{2}}{2\sigma^{2}}\right\}. \end{array}\right. \end{array}$$

The spatial error diffusion formula is the human visual modulation function MTF. The mathematical model expression of modulation transfer function is

(6) $$\begin{array}{c} \left\{\begin{array}{c} H_{f}\left(f_{r}\right)=2.6\left(0.0192+0.114f_{r}\right)\exp\left\{-{\left(0.114f_{r}\right)}^{2}\right\},\\ f_{r}=\sqrt{f_{x}^{2}+f_{y}^{2}}. \end{array}\right. \end{array}$$

In practice, there are many error diffusion methods, and the method that meets the requirements of good colour visual effect according to the actual effect is scientific and feasible. The filter *x* proposed in the error diffusion jitter table Floyd–Steinberg is a pixel value, and the gray-scale error generated by it will be dispersed to four adjacent pixels. In this filter, the sum of the numbers is 16. At this time, assuming that there is an error value between the gray value of the pixel and the black-and-white threshold, 7/16 of the error is added to the right pixel, 3/16 of the error is added to the lower left pixel of *X*, 5/16 of the error is added to the lower right pixel of *X*, and the remaining 1/16 of the error is added to the lower right pixel of *X*. For example: the gray level of the original image is 256, and the gray value of the upper point is 240 (0∼255). If you want to convert this image into 32 gray levels, the simplest method is to divide each pixel by 32, then the converted gray value is 240/32 = 7.5, and it is 7 after keeping the integer digits. In this way, the converted value has an error of 0.5. The simplest error diffusion method is to place the 0.5 error on the right/lower point of the point. We can distribute it to the right, lower right ,and lower points in the ratio of 3 : 2 : 3. That is, we add (0.5 *∗* 16) *∗* 3/8 = 3 to the right and lower points, and add (0.5 *∗* 16) *∗* 2/8 = 2 to the lower right points.

### 3.2. Image Colour Element Analysis Model

It is to classify the processed images and select the features to be extracted on the basis of segmentation. Some parameters are measured, then these features are extracted, and finally classified according to the measurement results. So, image recognition is to find out the shape, texture, and other features of each part after segmentation, that is, feature extraction sometimes includes image segmentation, so as to classify the image and analyze the structure of the whole image. In image recognition, there are several representative theories and methods: matching image recognition method, syntactic image recognition method, fuzzy image recognition method, and neural network image recognition method. This paper mainly relies on the CNN neural network for image colour analysis. The specific methods are as follows: considering that most of the data or tasks of image recognition are related, we can share the learned model parameters with the new model in some way through migration learning, so as to improve and optimize the learning efficiency of the model without learning from zero, so as to reduce the repeated workload and dependence on datasets. Inception-v3 model takes the convolutional neural network as the core. There are 5 convolution layers, 3 maxpooling layers, and 11 hybrid layers from input to output. The hybrid layer includes maximum pooling layer and average pooling layer. Convolutional neural network can be divided into input layer, hidden layer, and output layer. The structure of deep neural network is designed as shown in Figure 5:

The input layer preprocesses the data; the hidden layer includes convolution calculation, pooling, and excitation layers; the output layer outputs the calculation results. When training the inception-v3 model, extract the RGB values of all pixels of the original image and form three numerical matrices, which are input through three different channels and convoluted; during convolution calculation, in order to reduce the amount of calculation and ensure that the visual field of the image does not change, the convolution kernel is changed from 1 to 5 × 5 calculation conversion to 2 times 3 × 3. Calculation: after completing one convolution calculation, the convolution output data is used as the input data of the next operation. In the pooling layer, for the characteristic matrix with depth *D*, each layer is pooled separately. In the mixing layer, convolution and pooling are carried out synchronously to achieve efficient feature extraction so that the model has the characteristics of high efficiency and high accuracy. Using the method of transfer learning, the concept-v3 model is applied to the field of mineral image recognition. Using the pretraining model, the metamodel parameters can be used again to reduce the time cost.

### 3.3. Colour Component Analysis Based on Rotating Principal Component Analysis

In practical application, when the principal component analysis method is directly used to obtain the feature vector set a, it will face the problem of “negative index”, which makes the results have no practical significance. Therefore, the initial feature vector must be transformed into a set of feature vectors with clear meaning that can represent the actual basic colour components by linear transformation or geometric rotation. This transformation relationship must meet three important conditions: (1) the eigenvector obtained after rotation should be a set of fully positive vectors; (2) the elements in the rotated eigenvector should be differentiated into 0 or 1 by column; (3) the sum of variance in the direction of the transformed eigenvector should be the largest. The most commonly used transformation process is the so-called maximum variance orthogonal rotation method, that is, the rotating principal component analysis proposed in this paper. In the process of rotation, the principal component factor axis and load factor matrix (i.e. eigenvector set) always maintain rigid rotation. In the process of rotation transformation, an important problem worth considering is how to determine the number of principal components to be transformed. If the number is too small, the capacity of eigenvector bases will be too small to cover the original spectral space, which will affect the final accuracy of eigenvector reconstruction; the larger the number, the longer the operation time is required, and even the expected results that meet the above three conditions at the same time cannot be obtained. Therefore, the Gutt-man criterion is adopted in this paper, and only the principal components whose variance percentage is not less than 1% are processed by rotation transformation.

Given an *n* × *N* orthogonal matrix *T*, equation (3) can also be defined as the following form:

(7) $$\begin{array}{c} S\approx Af=\left(AT\right)\left(T^{T}f\right), \end{array}$$

where *AT* can be regarded as the load factor matrix corresponding to the new common factor or principal component *T*^*T*^*f* after orthogonal transformation, that is, the obtained eigenvector basis.

Rotate every two columns of a in turn, and a total of *n*(*n* − 1) transformations are required. After all rotations are completed, it is a cycle. The total variance of the square of the load factor of the original variable *s* on the new common factor *f*_*j*_, (*j*=1,2,…, *n*) is

(8) $$\begin{array}{c} V^{\left(1\right)}=\sum_{j=1}^{n}V_{j}^{\left(1\right)},\\ =\sum_{j=1}^{n}\left\{E\left({\left(a_{j}^{*2}\right)}^{2}-E{\left(a_{j}^{*2}\right)}^{2}\right)\right\},\\ =\sum_{j=1}^{n}\left\{\frac{1}{m}\sum_{i=1}^{m}{\left\{\frac{a_{ji}^{2}}{h_{i}^{2}}\right\}}^{2}-{\left\{\frac{1}{m}\sum_{i=1}^{m}\left\{\frac{a_{ji}^{2}}{h_{i}^{2}}\right\}\right\}}^{2}\right\}, \end{array}$$

where *h*_*i*_^2^ represents the total variance contribution rate of the new principal component *f*^*∗*^ to the variable *S*_*i*_, which can also be called the commonality of the variable *S*_*i*_, and *a*_*ji*_^2^ represents the variance contribution value of each new principal component *f*^*∗*^ to the variable *S*_*i*_. In equation (6), replacing *Aji* with *a*_*ji*_^2^ is to avoid the influence of negative load factor in the operation process, and dividing by *h*_*i*_^2^ is to eliminate the influence caused by the difference of common degree of each variable.

## 4. Simulation Results and Performance Analysis

### 4.1. Reliability of Principal Component Analysis

In this paper, Munsell matte collection I, which contains the reflection spectrum of 1,250 colour samples, is used as the experimental data. Each sample contains 61 elements. In order to meet the prerequisite of rotating principal component analysis, *E*(*S*)=*E*(*f*)=0, the original spectral measurement data are processed by central normalization, that is, *S*-*E* (*s*) is used to replace the original dataset *s* for principal component analysis. It can be proved that the central normalization of the original data set does not affect the structure of its covariance matrix.

After principal component analysis, the first four principal components are selected as the objects to be converted based on Guttman criterion, and their variance contribution rates to the original spectral space are 79.5%, 64%, 13.06%, 4.63%, and 1.18% respectively, and the contribution rate of cumulative variance was 98.51%. The minimum value selected here *ε* Equal to 10-8, when the total variance increment of the square of the relative load factor before and after cyclic treatment is less than *ε*, And when the new load factor matrix can be regarded as a set of full positive vector sets with values ranging from 0 to 1 (subject to normalized polarization processing), the rotation transformation processing can be stopped to obtain the final result.  Figure 6(a) shows the four original eigenvectors obtained by principal component analysis based on the normalized spectral data, and Figure 6(b) shows the four corresponding eigenvectors obtained after rotating principal component analysis, in which *EV*_*i*_ is the *i*th spectral spatial eigenvector. They represent the basic colour prediction components desired in this paper, and their cumulative variance contribution rate to the original spectral spatial information reaches 98.52%. By comparing Figures 6(a) and 6(b), it can be seen that the problem of “negative index” when directly using the principal component analysis method to obtain the feature vector set has been well solved after geometric rotation. According to Figure 6, it can be predicted that Munsell matte collection is composed of four basic colour blocks: red, green, blue, and purple. The prediction result is basically consistent with the actual colour components of Munsell matte collection.

### 4.2. Image Colour Element Management Performance Verification

In order to extract the image texture more accurately, the texture features can also be extracted according to the colour change of the surface. In this paper, the depth network is used to analyze the image colour. The parameters mainly include number of network layers, number of neurons in each layer, activation function ,and selection of training set. In computer vision, colours can be divided into 16777216 kinds, which can be obtained by arranging and combining the RGB values of the three primary colours. Therefore, to judge whether the colour of the mineral surface has changed, you only need to judge whether the proportion of RGB has changed. By inputting the image data of enhanced texture and setting inception-v3 as the pretraining model, the classification and recognition model of image element data can be trained. The length and width of the original input image of the model are set to 299. If the input image does not meet the requirements, the program will automatically cut and zoom so that the length and width of the image are 299; the colour image can be decomposed into RGB three colours, so the training depth of the model is set to 3; the bottleneck tensor of the model is a 2048-dimensional matrix, which is used to store the characteristics of the image. The softmax classifier is trained. The number of iterative steps of model training is 20000 and the learning rate is 0.01. During training, 100 images are randomly selected as the training set for each training 10 images randomly selected as the test set. When using the test set to verify the training results, the images in the training set cross verify each other so as to achieve the purpose of evaluating the model. The simulation results are shown in Figure 7. As shown in the figure, the preliminary analysis of image elements can be realized through the image colour and element model based on deep learning.

### 4.3. Comparative Simulation

In this paper, the modified model is solved in C language. The conversion accuracy of the modified model can be reflected in Table 1, and Figure 8 shows the verification results of 24 colour blocks with even colour sequence of neutral gray ladder rule superimposed by three colour dyes in *it*/2 colour target *Xb*, *Yb*, *Zb*, *Xq*, *Yq*, *Zq*, and Δ*E* represents the standard values of *x*, *y*, and *z*, the values of *x*, *y*, and *z* calculated by the correction model and the colour difference between them. Figure 8 is the statistical table of the conversion accuracy of all 288 colour blocks on the colour target by using the algorithm in this experiment, the polynomial fitting algorithm which is widely used and has relatively high conversion accuracy and the ordinary BP neural network algorithm.

It can be seen from the results in Table 1 and Figure 8 that the average colour difference between the *XYZ* calculated value obtained by the modified model in this paper and the *XYZ* standard value obtained by the standard database for the 288 colour samples tested Δ*E* ≤ 5 NBS, and the number of colour blocks with an error of more than 5 and the average conversion error obtained by this algorithm are significantly less than the conversion results of the polynomial fitting algorithm and the BP neural network algorithm. The colour difference unit is the colour difference unit adopted by the National Bureau of standards of the United States. According to the research results of colourimetry, generally when Δ*E* ≤ 5 NBS units, it can be considered as visual equivalent. Therefore, the horizontal and vertical comparison can show that the correction model proposed in this paper has satisfactory accuracy and can effectively analyze and manage image colour data according to various actual situations. The image colour element analysis algorithm proposed in this paper overcomes the defect that the commonly used algorithm does not consider the intermediate process of colour conversion and only controls the input and output values of sample colour blocks, which is difficult to ensure the conversion accuracy.

The experimental simulation in this paper is realized in the environment of MATLAB 7.0. In order to verify the effectiveness of this method, the size of 140 is selected × 140 Lena, car and fruit images. In order to further verify the adaptability of the algorithm, simulation verification is carried out. In the MATLAB simulation experiment, the RGB value of colour image is used to analyze the image colour elements. The model analysis results are shown in Figure 9. Experiments show the effectiveness of this method and improve the signal-to-noise ratio of the image.

## 5. Conclusion

Based on the deep learning theory and transfer learning method, combined with the physical properties of image intensity and colour, this paper extracts the colour and element features of 6,203 images, retrains the concept-v3 model based on the image of enhanced texture, builds a deep learning model system suitable for image element analysis and correction, and builds an image colour model by extracting colour features. Quantifying the colour difference of image reproduction, establish a model, and further establish a modified error diffusion model for better colour management and correction of map image analysis. The results are as follows: (1) using the colour correction algorithm of error diffusion model, the over corrected error diffusion method can maximize the diffusion of dot error, and the corrected error diffusion can preserve the image details, especially the details detected in the whole gray range, and restore the distribution naturally. (2) The depth learning algorithm is used to extract the colour features of the image, and the colour model is obtained. Combined with the depth learning model and colour feature model, the image element and colour recognition model are established. (3) In the process of colour reproduction, in order to achieve the ideal spectral matching effect, a new basic colour component analysis method based on rotating principal component analysis is adopted. It transforms the original feature vector into a set of all positive vectors representing the actual basic colour components by rotating and transforming it. Simulation results show the reliability and effectiveness of the algorithm. Due to the limitations of experimental conditions, the method proposed in this paper cannot carry out colour elements for low pixel images. The next step is to study the analysis of low pixel images.

## Figures and Tables

**Figure 1:** The structure of intelligent analysis of image colour data elements.

**Figure 2:** Isomerization tensorflow architecture based on docker container cluster.

**Figure 3:** Overall structure figure of image colour data element analysis algorithm based on neural network.

**Figure 4:** Visual error diffusion model.

**Figure 5:** Structure of deep neural network.

**Figure 6:** Rotating principal component analysis results. (a) Feature vector. (b) Positive vector.

**Figure 7:** The structure of improved sequential pattern mining algorithm.

**Figure 8:** The comparison results with other methods.

**Figure 9:** The comparison results under different image type.

**Table 1:** The structure of improved sequential pattern mining algorithm.

Number	*Xb*	*Yb*	*Zb*	*Xq*	*Yq*	*Zq*	Δ*E*
1	3.46	2.99	3.68	3.64	3.75	3.01	0.19
2	7.84	8.25	6.54	8.28	8.76	7.13	1.08
3	12.54	13.57	11.25	17.36	16.85	11.65	1.86
4	19.61	21.03	17.13	28.67	24.64	24.85	1.71
5	37.65	36.05	37.05	33.58	35.06	39.04	1.95
6	60.86	63.21	53.27	70.61	75.31	56.89	7.51

## Data Availability

The data used to support the findings of this study are available from the corresponding author upon request.
